RETRACTED

# The Effects of Positive or Neutral Communication during Acupuncture for Relaxing Effects: A Sham-Controlled Randomized Trial

**DOI:** 10.1155/2016/3925878

**Published:** 2016-02-11

**Authors:** Annelie Rosén, Mats Lekander, Karin Jensen, Lisbeth Sachs, Predrag Petrovic, Martin Ingvar, Anna Enblom

**Affiliations:** ^1^Department of Clinical Neuroscience, Osher Centre for Integrative Medicine, Karolinska Institute, 171 77 Stockholm, Sweden; ^2^Stress Research Institute, Stockholm University, 106 91 Stockholm, Sweden; ^3^Department of Medical and Health Sciences, Division of Physiotherapy, Linköping University, 581 83 Linköping, Sweden

## Abstract

*Introduction*. The link between patient-clinician communication and its effect on clinical outcomes is an important clinical issue that is yet to be elucidated.* Objective*. Investigating if communication type (positive or neutral) about the expected treatment outcome affected (i) participants' expectations and (ii) short-term relaxation effects in response to genuine or sham acupuncture and investigating if expectations were related to outcome.* Methods*. Healthy volunteers (*n* = 243, mean age of 42) were randomized to one treatment with genuine or sham acupuncture. Within groups, participants were randomized to positive or neutral communication, regarding expected treatment effects. Visual Analogue Scales (0–100 millimeters) were used to measure treatment expectations and relaxation, directly before and after treatment.* Results*. Participants in the positive communication group reported higher treatment expectancy, compared to the neutral communication group (md 12 versus 6 mm, *p* = 0.002). There was no difference in relaxation effects between acupuncture groups or between communication groups. Participants with high baseline expectancy perceived greater improvement in relaxation, compared to participants with low baseline levels (md 27 versus 15 mm, *p* = 0.022).* Conclusion*. Our data highlights the importance of expectations for treatment outcome and demonstrates that expectations can be effectively manipulated using a standardized protocol that in future research may be implemented in clinical trials.

## 1. Introduction

Most medical treatments may be divided into a specific treatment component, for example, a pharmacological substance, and a nonspecific component that includes the context surrounding the delivery of treatment [1]. The nonspecific treatment component is typically conveyed via treatment information and the patient-clinician interaction, and examples of these effects are seen in placebo studies. Expectancy is accepted as one of the key contributors of the placebo effect [2] and a wide range of studies of placebo treatments have elucidated pathways through which placebos can be activated, often described as an interaction between psychological processes (e.g., expectations, motivation, and hope) and neurobiological mechanisms (e.g., endocrine and immune functions) [3, 4].

RETRACTED

The communication between a patient and clinician may have significant effects on treatment outcomes [5, 6] and one likely mediator of the communication-related treatment effects is patient expectations, as demonstrated by placebo studies in various clinical domains [7, 8]. To investigate the link between patient-clinician interactions and patient expectancy in a clinical setting, acupuncture is suggested as an effective method [9–11], as acupuncture is a procedure with known nonspecific treatment components [12]. The specific treatment components of genuine acupuncture include skin penetration and needle manipulation [13, 14], which, according to Western acupuncture, are suggested to be the main mechanisms for producing treatment effects, for example, through stimulation of afferent nerves that modulate spinal transmission and brain processes [15]. However, it is not clear whether the specific characteristics of genuine acupuncture cause the positive effects on physiological functions, such as heart rate, blood pressure, and cortisol levels [14, 16–18], or if the same effects could be obtained from the nonspecific components of acupuncture, measured with a credible, nonpenetrating, sham procedure [19, 20]. In fact, studies often show no difference between genuine and sham acupuncture with respect to clinical outcomes [12, 21–23].

Several studies have demonstrated that the patient-clinician interaction can have large effects on treatment outcomes, indicating that the medical ritual that surrounds acupuncture may shape expectations and contribute to treatment outcomes [10, 23, 24]. Investigating the link between patient-clinician communication and patient expectancy has the potential to clarify important mechanisms that carry nonspecific treatment effects. Today, there is a lack of understanding of how clinicians contribute to patients' expectations regarding treatment outcome and to what extent this is clinically relevant. Is it possible to systematically influence expectations to improve treatment outcome? As a scene for investigating the importance of expectations on treatment outcomes, we used acupuncture for relaxation effects. It is commonly reported that participants experience a sense of relaxation during acupuncture treatment [25, 26], yet it is not known if the effects are related to the specific effects of needling or nonspecific effects associated with the treatment procedure [22, 27, 28].

RETRACTED

In the present study, the aim was to investigate the relationship between clinicians' verbal communication (positive or neutral) and the participants' treatment expectations in a placebo-controlled acupuncture study of relaxation. We investigated if clinicians' positive or neutral information about the treatment had an effect on (i) participants' expectations and (ii) short-term relaxation effects in response to genuine or sham acupuncture. In addition, we investigated if treatment expectations were related to outcome.

## 2. Materials and Methods

In this study, we used a randomized sham-controlled design, where the participants and study evaluator were blinded as to the randomization of acupuncture treatment and communication type, while the person performing the acupuncture was not blinded. The Regional Ethics Committee of Linköping, Sweden (Dnr 2013/80-31), approved the study and all participants gave written informed consent. The trial is registered at the US National Institutes of Health (ClinicalTrials.gov) # NCT02525445.

### 2.1. Participants and Therapists

Participants were consecutively recruited by nine therapists (Figure 1), either via personal communication or by using a written flyer regarding the study. Both the personal initial contact and the flyer contained the same information, that is, “we are conduction a study regarding acupuncture for relaxing effects-would you like to receive further information?” The participants were healthy individuals, mainly recruited from the therapists' networks in their local community. Prior to inclusion, participants were given written information and screened for inclusion criteria (minimum age 18 years, understanding and writing Swedish). Exclusion criteria included previous education in acupuncture therapy. The participants were informed that they would be randomized to one of two types of acupuncture needles: one that penetrated the skin and one where needles were placed against the skin. Participants were also informed that they would be randomized to two types of “treatment procedures” performed by the therapist, without further specification, as to prevent participants from knowing about the contents of the communication types. All therapists were registered physiotherapists and had formal education in acupuncture (comparable with 15 ECTS points) and experience of performing acupuncture (2 to 20 years).

### 2.2. Procedure

Expectation and relaxation measures were collected at three time points (*T*0–*T*2): two hours before treatment (baseline, *T*0) and directly before (*T*1) and after treatment (*T*2) (Figure 2). The treatment procedure lasted for approximately 30 minutes. Directly after *T*1, prior to treatment onset, a randomization table (computer generated) was used to allocate the blinded participants to (a) acupuncture treatment type (genuine/sham) and to (b) communication type (positive/neutral). The treatments were performed in an environment chosen by the participants and therapist, and the participants could sit or lie. The therapists were introduced to the standardized study protocol by practical demonstrations of the logistic steps, including the acupuncture types (genuine/sham) and the communication types (positive/neutral communication). The study evaluator (Annelie Rosén) was blinded as to the randomization until the analysis of the primary outcome was complete for each experimental group.

RETRACTED

### 2.3. Treatment Intervention: Acupuncture Types

*Genuine acupuncture* was administered in accordance with Western medical style (sharp needles diameter of 0.25 × length of 40 millimeters (mm)) bilaterally to the acupuncture point pericardium six (PC6) between the tendons of palmaris longus and flexor carpi radialis at two body-inches (one body-inch is approximately 1.5 cm) proximal to the wrist at 0.5-body-inch depth. The therapists manipulated the needles three times per treatment by rotating, thrusting, or lifting the needles. When the participant reported a sense of numbness or soreness and the therapist noted a minimal muscular contraction around the needle [19, 29], the therapist registered this as a “needle sensation” in a treatment protocol.

*Sham acupuncture* was administrated (blunt needles diameter of 0.25 × length of 40 mm) bilaterally to a nonacupuncture point four body-inches proximal to and one body-inch radial from the PC6, with the telescopic nonpenetrating Park's sham needle [20]. Park's credible needle looks identical to a real needle but glides upward into its handle, giving an illusion of penetration [19, 30]. A marking tube, identical for both acupuncture types, held the sham needle in place. The therapists manipulated the needles a few seconds three times per session until the needles touched the skin—but no “needle sensation” occurred—and then lifted the needles up from the skin [31]. Except for placing and manipulating the needle, the sham needle thus performed no pressure against the skin similar to the procedure in other studies [19, 20, 32].

### 2.4. Treatment Intervention: Verbal Communication Types

To manipulate the nonspecific component* expectation* during treatment, a standardized study protocol for the two verbal communication types was used, similar to a study by Suarez-Almazor et al. [24].

*The Positive Communication Type*. The therapist conveyed at least three out of several positive statements, such as the following: “Many acupuncture studies have shown excellent results concerning relaxation effects,” “Brain imaging studies show that acupuncture treatments affect areas that affect pulse, blood-pressure and muscle tension,” “I have had positive effects on relaxation with this treatment before,” and “Also in studies that investigated other effects of acupuncture than relaxation, the most common positive side effect was a sense of relaxation.”

RETRACTED

*The Neutral Communication Type*. The therapists conveyed at least three out of several neutral statements, such as the following: “During treatment you will just lie down and rest and I will not talk so much to you,” “We do not really know if acupuncture is a good method for relaxation effects; thus we need to perform this study,” “It is important for me to focus on the needling procedure; therefore I will not talk so much, it's not to be impolite to you,” and “One cannot know if you will experience relaxation effects of the acupuncture treatment, I have treated persons who thought differently about it.”

### 2.5. Data Collection

#### 2.5.1. Sociodemographic and Other Baseline Data

A baseline questionnaire included previously used [26] questions for sociodemographic data (e.g., gender and age) and earlier experience of (yes/no) and belief in (yes/no) the effect of acupuncture for 17 symptoms (e.g., pain). Health status was graded on the Swedish version 100 mm vertical EuroQol (EQ) Visual Analogue Scale (VAS), anchored with 100 (best imaginable health state) and 0 (worst imaginable health state) [33].

#### 2.5.2. Expectation and Relaxation Data

The participants rated their* expectancy *using questions adapted from our previous acupuncture studies [21, 26], “Do you believe that the needling treatment that you are going to receive is effective to provide relaxation/reduce muscle tension/reduce stress?” measured with a 100 mm VAS anchored with 0 (“Do not believe at all it's effective”) and 100 (“I completely believe it's effective”). The questions used the modified tempus “received” and “was effective” after treatment. To rate relaxation* per se*, participants rated relaxation, muscle tension, and stress using the previously used [26] question: “Do you feel relaxed right now?” measured with a 100 mm VAS anchored with 0 (“Not relaxed at all”) and 100 (“Completely relaxed”). The same question was asked for “muscle tension” and “stress.”

#### 2.5.3. Heart Rate and Blood Pressure

The therapists measured heart rate and blood pressure [34] with a digital wrist blood pressure monitor (König Electronic, HC-BLDPRESS11) before and after treatment. The participants placed their left arm relaxed on the surface with their palm up and the monitor was placed approximately 2 centimeters above the wrist joint.

RETRACTED

#### 2.5.4. Treatment and Blinding Data

The therapists registered their own compliance to the study protocol during the treatment sessions (variables shown in Table 1). After treatment, the participants gave binary answers to the blinding question “Do you think that you have been treated with needles that have penetrated the skin, or do you think the needles have been placed just against the surface of your skin?” [26] and the question “Do you think that you have received acupuncture by a therapist who emphasized the expected positive effects or not?” After each binary question, the participants graded “How sure are you about your answer?” (“Not sure at all, just guessed” and “fairly sure, entirely sure”). The participants graded the perceived needle-induced pain (“No/little/moderate/very painful”) and their interest in further acupuncture treatments (“No/little/moderate/very/completely interested”).

## 3. Statistical Methods

### 3.1. Primary Outcome and Sample Size

The primary outcome was the change in relaxation from the period before to that after treatment. To detect a clinical relevant difference of VAS 10-millimeter change [35, 36] between the genuine and the sham acupuncture type, or between the positive and the neutral communication types, we calculated that a total sample size of 208 participants was needed (80% power, significance level 0.05). A possible dropout rate of less than 20% was expected, ending up with a recruitment goal of 250 participants.

### 3.2. Statistical Analyses

For comparing the effect of the acupuncture and communication types, Mann-Whitney *U* tests were used for ordinal variables and *t*-tests for the continuous variables. For comparisons of the four acupuncture/communication group combinations, Kruskal-Wallis tests were used for ordinal variables. For categorical data, we used Chi square. For dependent within-group comparisons between the period before and that after treatment, Wilcoxon matched pairs test was used regarding ordinal variables. For investigating if different levels of baseline treatment expectations were related to outcome, we categorized the question “Do you believe that the needling treatment is effective to provide relaxation?” measured with a 100 mm VAS into three categories: low belief = 0–32 mm, moderate belief = 33–66 mm, and high belief = 67–100 mm. Data analysis was performed using SPSS (version 22.0). The significance level was set as *p* < 0.05, two-tailed.

## 4. Results

### 4.1. The Participants

We randomized 243 participants: 122 to genuine acupuncture (62 to positive and 60 to neutral communication) and 121 to sham acupuncture (60 to positive and 61 to neutral communication), between September 2013 and February 2014 (Figure 1). In the genuine acupuncture group, one participant never came to treatment and one participant interrupted treatment, leaving 241 participants completing the treatment session. A typical participant was 41.8 (mean, m) years old, married (74%), woman (76%), working in public sector (56%), with a baseline EQ-VAS health status of 79 mm, and without previous experience of acupuncture (55%) (Table 2).

RETRACTED

### 4.2. Baseline Characteristics

Participants' baseline characteristics did not differ between the acupuncture nor the communication groups (Table 2), regarding baseline measures of treatment expectancy (genuine versus sham, *p* = 0.705; positive versus neutral, *p* = 0.150), participant-reported relaxation (Figure 3), and objectively measured relaxation (Table 4). However, there were two exceptions. In the positive communication group, fewer participants had previously received acupuncture but believed in acupuncture as effective for a higher number of symptoms, compared to the neutral communication group (Table 2).

### 4.3. The Change in Expectations after the Therapists' Communication

Both the positive and the neutral communication group significantly increased their expectations of receiving relaxation from needling (*p* < 0.001) (Table 3). Participants (*n* = 119) who received needling by a positively communicating therapist had increased their expectations of relaxation effects from the needling more (median (md) 12 mm VAS, 25th–75th percentile (IQR) 2–22) than the participants (*n* = 111) who received needling by a neutrally communicating therapist (md 6 mm VAS, IQR −4–16), *p* = 0.002 (Table 3).

### 4.4. The Change in Participant-Reported Relaxation after Genuine or Sham Acupuncture

Both the genuine and sham acupuncture group improved their sense of relaxation and decreased subjectively rated stress and muscle tension after treatment compared to before treatment. There was no statistical difference in perceived relaxation, stress, or muscle tension between the acupuncture types (*p* = 0.428, *p* = 0.771, and *p* = 0.666, resp.) (Figure 3).

### 4.5. The Change in Participant-Reported Relaxation after Needling by a Neutrally or Positively Communicating Therapist

Both the positive and the neutral communication group significantly improved their sense of relaxation and decreased stress and muscle tension after treatment compared to before treatment. There was no statistical difference in perceived relaxation, stress, or muscle tension between the communication types (*p* = 0.256, *p* = 989, and *p* = 0.703, resp.) (Figure 3). When separating the communication types into the genuine and sham acupuncture type, the participants that received genuine acupuncture in combination with positive communication improved relaxation higher in absolute number of steps (md 27 mm VAS, IQR 10–45), as compared to participants that received genuine acupuncture in combination with neutral communication (md 18 mm VAS, IQR 2–36; *p* = 0.118).

RETRACTED

### 4.6. Expectations in relation to Change in Degree of Relaxation

Overall, participants with high baseline levels of expectations (i.e., expectation ratings 67–100 mm VAS; *n* = 81) to receive relaxation effects of the needling perceived greater improvement in relaxation (md 27 mm VAS, IQR 1–48) than participants with low expectations (i.e., expectation ratings 0–33 mm; *n* = 35) (md 15 mm VAS, IQR 2–36) (*p* = 0.046). After the therapists' communication during the needling, the participants having high beliefs in the effect of the needling (*n* = 136) also had greater improvements in relaxation (md 30 mm VAS, IQR 14–50) than the participants (27) with low belief in the effect of needling (md 5 mm VAS, IQR 0–21) (*p* < 0.001), irrespective of needle or communication group.

### 4.7. Blood Pressure and Heart Rate

After treatment, the genuine and the sham acupuncture groups did not differ in the size of decreased heart rate (*p* = 0.976), systolic blood pressure (*p* = 0.141), or diastolic blood pressure (*p* = 0.109), nor did the respective measures differ between the neutral and positive communication groups (*p* = 0.729, *p* = 0.161, and *p* = 0.088) (Table 4).

### 4.8. Blinding and Side Effects

The participants were successfully blinded, as 86% in the genuine acupuncture group and 72% in the sham group thought they had received a penetrating treatment (*p* = 0.008) (Table 1). Participants who believed they had received genuine acupuncture (*n* = 173) did not rate higher degrees of relaxation from the period before to that after treatment (md 23 mm VAS, IQR 8–46) than those who believed they had received sham acupuncture (*n* = 48) (md 25 mm VAS, IQR 9–56) (*p* = 0.400). Regarding communication type, a majority of the participants believed they received neutral communication during treatment (68%, Table 1).

Most participants in the genuine (88%) and in the sham group (98%) graded needle-induced pain as nonpainful or mildly painful. However, pain was reported more frequently in the genuine group (*p* < 0.001). Negative side effects were few and minor; the most common were feelings of numbness or tingling in the hand (24%) and bleeding around the needle (7%). One single participant fainted for a brief moment during sham acupuncture (Table 1).

RETRACTED

## 5. Discussion

Here we demonstrate that a verbal communication model could successfully affect expectations regarding effects of acupuncture, showing that positive communication led to increased treatment expectations. There was no difference in perceived relaxation between the genuine and sham acupuncture groups and the same was true for participants receiving positive or neutral communication. Participants with high levels of expectations at study entry perceived greater improvement in relaxation than participants with low expectations. Overall, our data illustrates significant effects of expectancy on outcomes, highlighting the complexity of expectations and treatment communication in acupuncture treatment.

The participants in the positive communication group had increased their expectations of relaxation effects more than the neutral group and were also more interested in receiving acupuncture for relaxation again. This indicates that a relatively brief verbal suggestion can be a successful method to enhance treatment expectations, with no added risks or harms. In spite of the difference in treatment expectancies between the communication groups, participants in the neutral communication group also displayed some degree of improved expectations. This is in line with previous knowledge demonstrating that “just being” in an intervention affects expectations towards a positive treatment outcome [1, 37, 38].

Overall, the perceived relaxation, reduced stress, and muscle tension improved from the period before to that after treatment, yet there was no difference between the genuine and sham acupuncture groups. Our results are consistent with other acupuncture studies, also failing to demonstrate differences between genuine and sham acupuncture [22, 26, 39]. In a recent systematic review [39], including 38 sham and genuine acupuncture trials for miscellaneous conditions, most studies (58%) reported no significant outcome differences and concluded that sham acupuncture may be as effective as genuine. The lack of difference in relaxation responses to genuine or sham acupuncture is a new finding, and, to the best of our knowledge, there are no other sham-controlled studies investigating relaxation effects of acupuncture. However, relaxing effects are a common positive side effect of acupuncture [25, 26] and in a recent study on cancer patients [26] we found that relaxation was the most prevalent positive side effect (58%), irrespective of genuine or sham acupuncture treatment.

In line with the lack of difference in relaxation effects between genuine and sham acupuncture, there was no difference in relaxation between the positive and neutral communication groups, even though participants in the positive group reported greater change in expectations. One explanation could be that expectations induced by verbal suggestions only account for part of the expectancy-driven effects on treatment outcomes. This is supported by the impact of baseline treatment expectations in our study, measured before any verbal suggestion took place. This suggests that baseline beliefs had a larger impact on treatment outcomes than experimentally induced verbal suggestions. In contrast to our results, a recent study [24] found that patients in a positive communication group had larger improvements in knee pain and satisfaction, compared to patients in a neutral group. Also, a seminal study by Kaptchuk and coworkers [10], investigating the effect of enhanced provider communication in patients with irritable bowel syndrome, found differences in the proportion of patients reporting adequate symptom relief, that is, 28% on waiting list, 44% in the “limited communication” group, and 62% in the “augmented communication” group. In our study, the lack of differences in degree of relaxation between the communication groups may be explained by the difficulty to obtain placebo effects in healthy participants [40, 41]. It is possible that healthy participants are less influenced by desire, motivation, and hope, which are factors known to mediate placebo effects [3, 42].

RETRACTED

Even though we did not find any significant differences between the communication groups, there was a trend towards larger increase in relaxation in the genuine acupuncture group with positive communication compared to the genuine acupuncture group with neutral communication (9 mm VAS difference between communication types). No similar difference was seen between the communication types during sham acupuncture.

Participants receiving positive communication were more likely to have interest in further acupuncture treatments, as 94% expressed interest in testing acupuncture again. This furthers the notion that our intervention significantly changed the mindsets of our participants. The finding bears clinical relevance, because a more positive attitude towards a treatment may increase treatment adherence.

Here, we found that participants with high treatment expectations at baseline had greater relaxation effects than participants with low baseline expectations. Also, participants' posttreatment reports of attributing the relaxation to the needling* per se* were associated with increased relaxation, irrespective of treatment or communication group.

Some sham-controlled acupuncture studies indicate that patients who believe they receive genuine acupuncture report larger treatment effects than patients who believed they received sham [43, 44]. Yet, in our study we found no differences in relaxation effects or expectations between participants who believed they had received genuine or sham acupuncture. Our results are in line with results reported by Kaptchuk et al. in an open-label placebo trial, where all participants knew they were on placebo treatment [45] but still displayed significant treatment effects. Altogether, these findings suggest that the healing mechanisms of placebo, which are largely affected by treatment expectations, are not always dependent on deception.

RETRACTED

This study did not find any differences between acupuncture groups or communication groups regarding objective measurements of blood pressure and heart rate. The same was reported for objective outcomes in a review investigating the effects of expectations in acupuncture studies; however only three studies in the review included objective outcome variables [8].

In order to isolate the specific versus nonspecific components of acupuncture treatment, we employed a design that compared genuine and sham acupuncture [19, 30]. It is essential that the sham device is able to successfully blind the treated participants and, if possible, the therapists too [46]. In our study, most participants (79%) believed they received genuine acupuncture, and in the sham group 72% believed they received genuine acupuncture, which indicates successful blinding. With the Park sham device, used in the present study, there is no blinding of the therapist, which prevented us from using a double-blind design. However, the outcome assessor (Annelie Rosén) was blinded to treatment allocation until after analyses of the primary outcomes, which decreases the risk of bias in our statistical analysis.

Furthermore, including nonnaïve participants in acupuncture studies may affect outcomes [27]. We included participants with previous experience of acupuncture treatment, as this would strengthen the generalizability. Conversely, there is a risk of interfering with the needle blinding, as participants with previous experience may know what genuine needling feels like. Although 44% of the participants in the sham group had previous experience of acupuncture, the blinding to needle type or perceived degree of relaxation was not affected. Our results further the importance of using a credible sham control, not only for evaluating the blinding success, but also to investigate if the participants' perception of treatment allocation affects outcome.

We used acupuncture effects on relaxation as a model to assess two key aspects of acupuncture treatment: firstly, to investigate the feasibility of changing treatment expectations by means of manualized verbal communication and, secondly, to study the specific acupuncture effects during genuine acupuncture compared to sham acupuncture. Hence, our study was not primarily designed to demonstrate the actual effect of needling on relaxation, since no natural history control was included. This means that, despite the majority of participants perceiving more relaxation after treatment, it cannot be excluded that improvements were partly explained by spending 30 minutes in a restful environment, in combination with the extra attention from the therapist.

RETRACTED

In sum, our data highlight the importance of expectations for treatment outcomes in acupuncture and demonstrate that expectations can be effectively manipulated using a standardized treatment protocol. Therefore, the present study may serve as a model for reinforcing treatment expectations in clinical trials in the future. As the present study included healthy participants, the model should be validated in clinical populations, where treatment expectations are thought to play an important role for boosting clinical effects.

## Figures and Tables

**Figure 1:** Inclusion and treatment of participants receiving acupuncture (genuine or sham) and communication (positive or neutral).

**Figure 2:** Schematic representation of the treatment procedure. The different time points (*T*) for measurements were two hours before treatment (baseline, *T*0), directly before treatment (*T*1), and after treatment (*T*2). The text boxes above the timeline represent data types collected at the different time points. Text boxes below the timeline represent time points and experimental events. The positive and neutral communication was performed between needle insertion and needle removal.

**Figure 3:** Relaxation status. Grade of relaxation, stress, and muscle tension (median) before and after treatment with genuine or sham acupuncture (a) performed by a positively or neutrally communicating therapist, (b) measured with a Visual Analogue Scale (VAS): from 0 = not at all to 100 = most possible. ^*∗∗*^ *p* < 0.001, significant difference between groups, comparing pre- and posttreatment values within groups.

**Table 1:** Blinding statements and genuine and sham acupuncture treatment related variables.

Variable	Total	Genuine acupuncture	Sham acupuncture	*p* value	Positive communication	Neutral communication	*p* value
Blinding, *n* (%)	*n* = 235	*n* = 118	*n* = 117	0.008^*∗*^	*n* = 118	*n* = 117	0.104
Penetrating the skin	185 (79)	102 (86)	83 (72)		98 (83)	87 (74)	
Placed against the skin	50 (21)	17 (14)	33 (28)		20 (17)	30 (26)	
How sure, needle type, *n* (%)	*n* = 236	*n* = 116	*n* = 117	0.001^*∗*^	*n* = 119	*n* = 117	0.128
Not sure at all	35 (15)	11 (10)	24 (20)		14 (12)	21 (18)	
Fairly sure	111 (47)	50 (43)	61 (52)		55 (46)	56 (48)	
Entirely sure	90 (38)	55 (47)	32 (26)		50 (42)	40 (34)	
Did the therapist emphasize the expected positive effects, *n* (%)	*n* = 235	*n* = 117	*n* = 118	0.547	*n* = 118	*n* = 117	0.000^*∗*^
Yes	76 (32)	36 (30)	40 (34)		58 (49)	18 (15)	
No	159 (68)	82 (70)	77 (66)		60 (51)	99 (85)	
How sure, commun. type, *n* (%)	*n* = 235	*n* = 117	*n* = 118	0.250	*n* = 118	*n* = 117	0.305
Not at all	26 (11)	14 (12)	12 (10)		15 (13)	11 (9)	
Fairly sure	125 (53)	56 (47)	69 (59)		64 (54)	61 (52)	
Entirely sure	84 (36)	48 (41)	36 (31)		39 (33)	45 (39)	
Needle-induced pain, *n* (%)	*n* = 239	*n* = 119	*n* = 119	0.000^*∗*^	*n* = 119	*n* = 120	0.725
Not painful	150 (63)	60 (50)	90 (75)		76 (64)	74 (62)	
Mildly painful	74 (31)	47 (39)	27 (23)		36 (30)	38 (32)	
Moderately painful	13 (5)	11 (9)	2 (2)		5 (4)	8 (6)	
Very painful	2 (1)	2 (2)	—		2 (2)	0 (0)	
Flush around needle points, *n* (%) of participants	*n* = 242		*n* = 121	1.0	NA	NA	
Yes	73 (30)	36 (30)	37 (31)				
No	169 (70)	85 (70)	84 (69)				
Side effects, *n* (%) of participants					NA	NA	
Bleeding, around needle points	*n* = 242	*n* = 111	*n* = 121	0.001^*∗*^			
Yes	17 (7)	15 (12)	2 (2)^b^				
No	225 (93)	106 (88)	119 (98)				
Numbness, tingling in the hand	*n* = 241		*n* = 120	0.000^*∗*^	NA	NA	
Yes	57 (24)	43 (36)	14 (12)				
No	184 (76)	78 (64)	106 (88)				
Dizziness	*n* = 241		*n* = 120	0.684	NA	NA	
Yes	6 (3)	4 (3)	2 (2)				
No	235 (97)	117 (98)	118 (98)				
Fainting	*n* = 241	*n* = 121	*n* = 120	0.498	NA	NA	
Yes	1 (1)	0 (0)	1 (1)				
No	240 (99)	121 (100)	119 (99)				
Tiredness	*n* = 241		*n* = 120	0.630	NA	NA	
Yes	61 (25)	29 (24)	32 (27)				
No	180 (74)	92 (76)	88 (73)				
Needle sensations, in number of treatments/total number of treatments		117/119	1/121^a^		NA	NA	
Numbers of needle sensations		*n* = 119	*n* = 121		NA	NA	
md (25th–75th percentile)		6 (5-6)	0 (0-0)				
Future interest in acupuncture treatment, *n* (%)	*n* = 234	*n* = 115	*n* = 119	0.337	*n* = 118	*n* = 116	0.008^*∗*^
Completely/much	174 (74)	81 (70)	93 (80)		96 (81)	78 (67)	
Moderately	34 (15)	22 (19)	11 (9)		15 (13)	19 (16)	
Little/not at all	26 (11)	13 (11)	13 (11)		7 (6)	19 (17)	

Number (*n*) and proportion (%) of participants are presented. NA = not applicable; communication types were not compared regarding these variables. ^a^The therapist used wrong needle by mistake once. ^b^Needle scratched the skin. ^*∗*^Statistical significant difference between groups.

RETRACTED

**Table 2:** Characteristics of the treated participants in the acupuncture and communication groups.

Characteristics	Total	Genuine acupuncture	Sham acupuncture	*p* value	Positive communication	Neutral communication	*p* value
Sex, *n* (%)	*n* = 238	*n* = 121	*n* = 117	0.448	*n* = 122	*n* = 116	0.409
Man	58 (24)	32 (26)	26 (22)		27 (22)	31 (27)	
Female	180 (76)	89 (74)	91 (78)		95 (78)	85 (73)	
Age in years: m ± SD	41.8 ± 13.2	42.7 ± 13.1	40.9 ± 13.6		40.5 ± 13.0	43.1 ± 13.6	0.132
Education, *n* (%)	*n* = 238	*n* = 120	*n* = 119	0.790	*n* = 121	*n* = 117	0.670
High school	4 (2)	3 (2)	1 (1)			4 (3)	
College	78 (33)	39 (33)	39 (33)		44 (36)	34 (29)	
Graduate school or higher education	156 (65)	78 (65)	78 (66)		77 (64)	79 (68)	
EQ-VAS score, (0–100)	*n* = 230	*n* = 116	*n* = 114		*n* = 116	*n* = 114	
md (25th–75th percentile)	80 (70–90)	80 (70–90)	80 (70–90)	0.665	81 (74–90)	80 (70–90)	0.141
Earlier experience of acupuncture treatment, *n* (%)	*n* = 225	*n* = 120	*n* = 118	0.687	*n* = 121	*n* = 117	0.039^*∗*^
Yes	108 (45)	56 (47)	52 (44)		47 (39)	61 (52)	
No	130 (55)	64 (53)	66 (56)		74 (61)	56 (48)	
Belief in acupuncture for at least one symptom^1^, *n* (%)	*n* = 232	*n* = 116	*n* = 116	1.000	*n* = 117	*n* = 115	0.284
Yes	216 (93)	108 (93)	108 (93)		111 (95)	105 (91)	
No	16 (7)	8 (7)	8 (7)		6 (5)	10 (9)	
Belief in acupuncture, number of symptoms^1^, m ± SD	*n* = 232	*n* = 115	*n* = 116		*n* = 117	*n* = 114	
	7.7 ± 4.7	8.3 ± 5.0	7.1 ± 4.3	0.060	8.4 ± 4.8	6.9 ± 4.4	0.013^*∗*^

Number (*n*) and proportion (%) of participants are presented. md = median, m = mean, SD = standard deviation, and EQ-VAS = Euro Qul Visual Analogue Scale. ^1^Out of maximum 17 different symptoms. ^*∗*^Statistical significant difference between groups.

**Table 3:** The participants' change in belief to receive relaxation effects (from pre- to posttherapy).

	Pretherapy: belief in relaxation effects	Posttherapy: belief in relaxation effects	Change: belief in relaxation effects	*p* value
Positive communication	*n* = 120	*n* = 120	*n* = 119	
md (IQR)	60 (39–74)	76 (59–89)	12 (2–22)	0.000^*∗*^
Neutral communication	*n* = 114	*n* = 116	*n* = 111	
md (IQR)	55 (40–72)	61 (40–83)	6 (−4–16)	0.000^*∗*^

Number (*n*) of participants; md = median; IQR = 25th–75th percentile. Expectations measured with Visual Analogue Scale (VAS) 0–100 mm from “Don't believe at all it's effective” to “I completely believe it's effective.” ^*∗*^Statistical significant difference between groups.

**Table 4:** The pretreatment levels and change between pre- and posttreatment in heart rate and blood pressure in the acupuncture and communication groups.

	Genuine acupuncture	Sham acupuncture	*p* value	Positive communication	Neutral communication	*p* value
Pretreatment, m ± SD						
	*n* = 120	*n* = 118		*n* = 122	*n* = 116	
Heart rate	68.1 ± 13.2	67.3 ± 10.3	0.607	67.9 ± 13.1	67.5 ± 10.3	0.788
	*n* = 119	*n* = 118		*n* = 122	*n* = 115	
Systolic blood pressure	125.1 ± 19.8	124.1 ± 19.6	0.694	125.4 ± 19.5	123.7 ± 19.9	0.501
Diastolic blood pressure	74.6 ± 10.0	74.5 ± 10.2	0.967	74.9 ± 10.0	74.2 ± 10.2	0.556
Posttreatment, m ± SD						
	*n* = 119	*n* = 118		*n* = 122	*n* = 115	
Heart rate	65.2 ± 10.2	64.4 ± 9.5	0.535	65.2 ± 9.8	64.3 ± 9.8	0.470
Systolic blood pressure	125.1 ± 19.8	124.1 ± 19.5	0.694	125.4 ± 19.5	123.7 ± 19.8	0.501
Diastolic blood pressure	74.5 ± 10.3	72.6 ± 9.5	0.145	73.0 ± 10.2	74.2 ± 9.6	0.363
Change in m ± SD						
	*n* = 119	*n* = 118		*n* = 122	*n* = 115	
Heart rate	−2.8 ± 8.8	−2.9 ± 7.6	0.894	−2.6 ± 8.8	−3.0 ± 7.5	0.729
	*n* = 118	*n* = 118			*n* = 114	
Systolic blood pressure	−1.5 ± 13.5	−3.4 ± 12.7	0.279	−3.6 ± 14.1	−1.2 ± 11.9	0.161
Diastolic blood pressure	−0.2 ± 8.5	−1.8 ± 7.7	0.107	−1.9 ± 8.5	−0.1 ± 7.6	0.088

Numbers (*n*) of participants; m = mean; SD = standard deviation.
